# Primitive Neuroectodermal Tumor of the Pancreas: A Case Report and Review of the Literature

**DOI:** 10.1155/2015/276869

**Published:** 2015-05-26

**Authors:** Uirá Teixeira, Marcos Goldoni, Michelle Unterleider, João Diedrich, Diogo Balbinot, Pablo Rodrigues, Rodolfo Monteiro, Daniel Gomes, José Sampaio, Paulo Fontes, Fábio Waechter

**Affiliations:** Gastrointestinal and Hepato-Pancreato-Biliary Surgical Division, Federal University of Health Sciences of Porto Alegre/Santa Casa Hospital of Porto Alegre, 91410-000 Porto Alegre, RS, Brazil

## Abstract

Primitive neuroectodermal tumors (PNETs) are presented as rare malignant neoplasms. In unusual cases, those neoplasms may arise in solid organs containing neuroendocrine cells, such as the pancreas. Herein the case of a 28-year-old patient that underwent gastroduodenopancreatectomy after the diagnosis of a huge mass (PNET) located in both head and body of the pancreas is reported. This is the 19th case of pancreatic PNET reported in literature.

## 1. Introduction

Primitive neuroectodermal tumors (PNETs) are presented as rare malignant neoplasms, showing different degrees of differentiation. They are often classified as small round cell tumors arising from soft tissues. PNETs also integrate Ewing's sarcoma family of tumors (ES), which represents 1% of all sarcomas [1, 2].

In rare cases, PNETs may arise in solid organs containing neuroendocrine cells, with previous reports on kidneys, urinary bladder, ovaries, uterus, parotid glands, heart, and lungs [3]. Besides these organs, the pancreas can also develop this type of tumors [3]—which accounts for 0.3% of the primary pancreatic neoplasms [4, 5]. Except for the case discussed here, only 18 other occurrences of pancreatic PNETs were previously reported in the world's literature.

These neoplasms occur predominantly in pediatric and teenaged populations [3], in a rate of 6.5 per million in patients up to 14 years [1]. They also present an insidious onset and often asymptomatic or poorly symptomatic course, even in advanced stages [4, 5].

A proper integration of the pathological, clinical, immunohistochemical, and cytogenetic findings is necessary for a successful diagnosis of pancreatic PNETs and also for distinguishing this group from other neoplasms with similar presentations [4]. Despite its rarity, this type of neoplasm must be considered in differential diagnosis when searching for pancreatic masses, especially in patients under 35 years of age [6].

In spite of the poor prognosis, surgical treatment followed by chemotherapy or radiotherapy or both is the most widely accepted option, given the aggressiveness of such neoplasms [4]. This is the case report of a 28-year-old patient that underwent surgery after PNET diagnosis, located in both head and body of the pancreas.

## 2. Case Report

A 28-year-old female patient was admitted to the Emergency Department of Santa Casa Hospital in Porto Alegre, Brazil. She was referring epigastric pain for 14 days, with partial relief due to the use of weak analgesics. The pain was associated with diffuse cutaneous pruritus, jaundice, choluria, and acholia.

On physical examination, the patient was in a good general condition, jaundiced, with a hardened palpable mass in the epigastric and right hypochondrium regions. Laboratory tests showed a cholestatic pattern (Table 1). Tumoral markers (CEA and CA19-9) were normal.

Initially, an abdominal ultrasonography was performed, revealing a voluminous heterogeneous hypoechoic mass measuring about 13 cm width, 9 cm length, and 13 cm height. It presented cystic areas inside, between left hepatic lobe and pancreas. It was not possible to determine the origin of the mass. Dilatation of intrahepatic bile ducts and proximal common bile duct was also referred to (Figure 1).

Computerized tomography with intravenous contrast unfolds a voluminous expansive lesion in pancreatic head and body, with well delimited borders, measuring about 12.8 × 12.1 × 10.9 cm. A heterogeneous density due to the presence of both liquid and solid areas is also shown in the CT. The image showed intense enhancement of an intravenous contrast agent. The lesion displaced adjacent structures, although no infiltration was detected. A significant ectasia of the intrahepatic and extrahepatic bile ducts could also be seen (Figure 2).

The patient was evaluated by the hepatopancreatobiliary team and underwent a gastroduodenopancreatectomy, performed uneventfully. The gross appearance of the lesion was a solid cystic mass, was encapsulated and multiloculated, and was with necrotic aspect areas, measuring a total of 11.5 cm along its longest axis (Figure 3).

The pathological study revealed a neoplasm of small round blue cells with scant cytoplasm arranged in nests with fibrovascular stroma. Few mitosis pictures and several areas of necrosis were also found. Immunohistochemistry was strongly positive for CD99 (Figure 4), vimentin, automated CKM (creatine kinase, muscle), and CD56. Furthermore, it was negative for antibodies present in neuroendocrine tumors (chromogranins, synaptophysin, and neuroblastoma), myogenin, automated CD10, *β*-catenin, automated RP (ribosomal protein), and LCA (leucocyte common antigen).

The patient recovered well postoperatively, presenting normalized levels of bilirubin, alkaline phosphatase, *γ*-glutamyl transpeptidase, aspartate aminotransferase, and alanine aminotransferase. She was discharged on the 13th day after surgery and remains well, without signs of recurrence after 3 years. Considering R0 resection and controversies in the literature, adjuvant treatment with chemotherapy and/or radiotherapy was not performed.

## 3. Discussion

Primitive neuroectodermal tumors (PNETs) represent about 1% of all sarcomas and have a five-year survival rate of approximately 50% [1–3, 7]. There are rare cases in which PNETs develop in solid organs [3, 8] arising, mainly, in soft tissues of the toracopulmonar region, pelvis, and lower limbs of children and young adults [3]. In organs containing neuroendocrine cells as the pancreas such kind of tumor is especially rare, accounting for 0.3% of primary tumors. [3, 4, 9, 10].

Histologically, the ES family of tumors is made of small monomorphic round cells with small nuclei and scant cytoplasm; nonetheless, there is a large group of tumors with the same pattern [2, 11]. What determines the familiarity between PNETs and ESs is the presentation, in both, of the same cytogenetic change. This change is seen in most of their malignant cells and consists of the characteristic chromosomal translocation t(11; 22) (q24; 12) [2, 3, 5, 11–13]. More than 90% of the ES/PNET shows this specific and reproducible translocation that evolves with variable degrees of differentiation. This is a reason for many authors to suggest that ES/PNET family is, actually, the same tumoral cell in different ends of the spectrum of differentiation [2, 6, 11, 12, 14].

An association of pathological, immunohistochemical, clinical, and cytogenetic features is, therefore, required for diagnosing pancreatic PNETs [4]. Furthermore, pancreatic PNETs must be included in the differential diagnosis of tumors containing small undifferentiated or poorly differentiated cells, neuroendocrine carcinomas, and pancreatoblastomas, among others [3, 6, 10].

Immunohistochemistry is extremely useful in diagnosing this neoplasm, as peripheral primitive neuroectodermal tumors substantially express a cell surface glycoprotein. This glycoprotein is product of the MIC2 gene (a pseudoautosomal gene located on the short arm of the X and Y chromosomes of PNETs and ESs cells), also called CD99 or p30/32_MIC2_, which is considered important in cell adhesion [2, 3, 6, 15].

Regarding the clinical presentation, it can be said that there is no specific set of symptoms for pancreatic PNETs. The onset of the disease seems to be insidious and producing few symptoms, with abdominal pain during palpation of the mass being the most referred to symptom. Mao et al. [4] indicate that patients tend to present jaundice, occurring mainly as obstructive jaundice; high gastrointestinal bleeding and severe anemia are also possible. Additionally, a unique case of hyperglycemia was reported by Mao et al.

Bose et al. [16] pointed out that, among 16 patients reported with ES/pancreatic PNET, 10 referred to abdominal pain as the most common symptom, with or without other symptoms. Moreover, jaundice was present in the diagnosis of 5 cases; 2 children (both females) were affected by precocious puberty, as well as 2 other cases with iron deficiency anemia secondary to gastrointestinal bleeding.

Among imaging tests, abdominal CT and MRI are the most used in the detection of these tumors. The diagnosis is not easy, as there is no pattern of radiological findings. The commonly found one, however, consists of masses with clear margins in the head of the pancreas [4, 12].

Discussing again the compilation of 16 patients of Bose and colleagues [16], 10 of these cases had findings in pancreatic head. In one of them, the tumor developed from the uncinate process and subsequently reached the head. Masses between 3 and 15 cm were reported. The authors also pointed to a variety of diagnostic modalities, where, nonetheless, CT is the most common. In one case recurrence in OctreoScan was found. Lymph nodes or other viscera involvement was observed in 3 patients.

The PNETs are characteristic aggressive tumors. Studies have shown that 25–30% of patients presented metastasis at diagnosis of PNET and it is believed to be an even larger number of patients with micrometastasis [2, 11, 12]. The most usual metastatic sites are lung, bone, and bone marrow. Because of this metastatic power, the association of chemotherapy with adequate local control by surgery or radiotherapy is prioritized. There is a trend of surgical treatment in most centers, even though it is not clear in the literature which method would give a better control of the primary tumor [2, 6, 12, 13]. The prognostic factors are, however, controversial. Ahmad et al. [17] analyzed 24 patients with extra skeletal Ewing's sarcoma and concluded that tumor size and metastatic disease are not significant factors for prognosis but age and surgical treatment are. de Alava and Gerald [2], in turn, claimed that the most important factor of poor prognosis is the presence of tumor dissemination at the time of the diagnosis.

Moschovi et al. [18] reported that the overall survival rate of patients with ES/PNET has progressively improved as a result of an effective systemic treatment and adequate resection and radiation for local control. Furthermore, the research suggested that multiagent intensive chemotherapy before surgery can further improve the prediction of these tumors.

Movahedi-Lankarani et al. [3] reported two cases of patients undergoing chemotherapy after Whipple procedure. One patient's survival was of 33 months with no evidence of recurrence, while the other relapsed and died four years after diagnosis. A third patient effectively treated with vincristine, doxorubicin, and cyclophosphamide was disease-free after 43 months. Perek et al. [19] reported the case of a man who underwent three surgical procedures associated with first, second, and third lines of chemotherapy for metastatic PNET, getting one of the largest known global survival, 50 months.

In spite of being an extremely rare disease, pancreatic PNETs should be considered in the differential diagnosis of pancreatic mass research, especially in patients younger than 35 years. Cases with undifferentiated small cell carcinoma, pancreatoblastoma, neuroendocrine carcinomas, and pancreatic endocrine tumors should also be investigated for PNETs. The clinical presentation of the tumor is diffuse and its histological findings are not exclusive. Most patients have a rapid growth mass, with nonspecific clinical symptoms and, often, abdominal pain.

These tumors present themselves as highly aggressive tumors with almost inevitable recurrence and metastasis, which makes the overall five-year survival rate reach almost 50%. Despite significant advances in treatment, there is still no definitive conclusion on which is the best therapeutic strategy at the moment.

## Figures and Tables

**Figure 1:** Abdominal ultrasonography showing a huge heterogeneous mass.

**Figure 2:** Abdominal CT reveals a voluminous lesion in pancreatic head and body (arrow).

**Figure 3:** Surgical specimen.

**Figure 4:** Small round cells with scant cytoplasm; immunohistochemistry was positive for CD99.

**Table 1:** Laboratorial findings.

Total bilirubin	4 mg/dL
Direct bilirubin	3,1 mg/dL
Alkaline phosphatase	319 U/L
Gamma-glutamyl transpeptidase	136 U/L
Glutamic-oxaloacetic transaminase	371 U/L
Glutamic-pyruvic transaminase	759 U/L
CA19-9	2,9 U/mL
CEA	3,0 ng/mL
